RETRACTED

# The Effects of Yoga Exercise on Pelvic Floor Rehabilitation of Postpartum Women

**DOI:** 10.1155/2022/1924232

**Published:** 2022-01-25

**Authors:** Qunfeng Li

**Affiliations:** ^1^Guangdong Polytechnic of Science and Technology, Zhuhai 510640, Guangdong, China; ^2^Macau University of Science and Technology, Macau, Taipa 999078, Macao SAR, China

## Abstract

Rehabilitation of the pelvic floor after delivery is very important for women. Pelvic floor rehabilitation can speed up the recovery of the postpartum vagina and pelvic floor muscle tension and elasticity and have a good effect on the prevention and treatment of postpartum vaginal prolapse and relaxation, urinary incontinence and other pelvic floor disorders. Thus, this article focuses on yoga exercise to explore its impact on postpartum pelvic floor rehabilitation. This article uses electrical stimulation and the treatment of pelvic floor muscles combined with the posture recognition algorithm, the yoga rehabilitation training program that has the best effect on the parturient is obtained, and the yoga myoelectric stimulation combined method and the traditional myoelectric stimulation method are designed for comparison experiments. The experimental results show that the parturients who have undergone the combined method of yoga myoelectric stimulation, in the resting state, contraction state, and Valsalva state, the position of the bladder meridian, the position of the uterus, and the position of the rectal ampulla of the parturient have a significant recovery compared those who have undergone the traditional electromyography treatment. In addition, the average area of hiatus in the pelvic floor ultrasound examination in the control group 42 days postpartum was 12.2605 cm^2^, while the average area of the hiatus in the pelvic floor ultrasound examination in the experimental group 42 days postpartum was 10.788 cm^2^; the average area of hiatus in the pelvic floor ultrasound examination in the control group at 3 months postpartum was 11.4805 cm^2^, and the average area of hiatus in the pelvic floor ultrasound examination in the experimental group at 3 months postpartum was 8.9475 cm^2^. To sum up, yoga had a very significant improvement on the physical indicators and mental health of postpartum women.

## 1. Introduction

Pelvic floor muscles refer to the group of muscles that close the bottom of the pelvis, mainly the levator ani muscle, which is an important part of the pelvic floor support tissue and is mainly composed of type I muscle fibers and type II muscle fibers [1]. It is attached to the bottom of the pelvis in a staggered manner and works with ligaments and other tissues to fix the bladder, uterus, and rectum in the pelvic cavity, and the urethra, vagina, and rectum pass through the pelvic floor tissue. Therefore, the pelvic floor tissue plays a vital role in supporting the pelvic organs such as the uterus, bladder, and rectum and maintaining female excretion, reproduction, sexual behavior, and other functions [2]. How to effectively treat postpartum pelvic floor muscle-related diseases is the focus of this article.

RETRACTED

In recent years, with the opening of the family planning policy, the research on pelvic floor health of postpartum women has continued to increase. As an important part of the pelvic floor tissue, the pelvic floor muscle has become an important research object of scientific researchers. Therefore, this article studies a method that combines yoga and electromyography to treat postpartum pelvic floor rehabilitation.

In the current environment of pursuing a healthy life, people are paying more and more attention to postpartum physical rehabilitation, and as the advantages of yoga exercise are put forward, more people are involved in the research of yoga exercise in postpartum pelvic floor rehabilitation [3, 4]. Dunleavy et al. designed a quasirandomized parallel controlled study and set up a community, university, and private clinic environments in four locations. 56 CNP participants scored ≥3/10 individuals over 3 months on the Digital Pain Rating Scale (control group *n* = 17, Pilates *n* = 20, yoga *n* = 19) [5]. Intervention exercise participants completed 12 group meetings, which were revised and progressed under the supervision of a physical therapist [6]. The Cheung C study compared the effects of Hatha Yoga (HY) and aerobic/strength training (ASE) on knee OA. He used a three-group design of randomized controlled trials: HY, ASE, and educational control. At baseline and 4^th^ and 8^th^ weeks, standardized instruments were used to measure OA symptoms and physical function; m-line is based on the intention to treat and adjusted to the baseline value [7]. Park and Kim studied mental health, fear of falling, and quality of life. The main analysis of the difference from the base determined the relationship between yoga coach image, nonverbal communication, coach trust, and intimacy of yoga center yoga practice participants. The results show that image has a positive effect on the subfactors of coach trust (sincerity, ability, consistency, altruism, and openness). Secondly, the subfactors (attitude, consciousness, profession, and role) of yoga coach image have a positive influence on intimacy [8]. Bhatia believed that yoga and physical exercise have been used as auxiliary interventions for cognitive dysfunction in schizophrenia (SZ), but there is no comparative comparison. The study passed a single-blind randomized controlled trial to evaluate whether yoga training or physical exercise training is based on previous preliminary research to enhance the cognitive function of SZ. According to preliminary research, the main outcome measure is the speed index of the attention cognition field in the computerized neurocognitive battery of the University of Pennsylvania [9]. The above-mentioned documents mainly discuss the importance of yoga exercise in the current environment where everyone is pursuing health. However, there are very few studies on the influence of yoga on postpartum pelvic floor rehabilitation. Basically, it can be said that there is no knowledge in this area. Therefore, in the actual writing of the thesis, this article needs to combine research and analysis on postpartum pelvic floor rehabilitation; it can also effectively improve maternal physical indicators and mental health.

RETRACTED

The innovation of this article is to understand the treatment methods of pelvic floor muscle clusters and combine them with the recognition of yoga asanas through asana recognition algorithms to obtain a new type of yoga training method that is very helpful for maternal postpartum pelvic floor rehabilitation. This method can effectively recover the position of the bladder meridian, the position of the uterus, the position of the ampulla of the rectum, and the area of the hiatus in the pelvic floor of the parturient.

## 2. Yoga Postpartum Pelvic Floor Rehabilitation Methods

### 2.1. Yoga Improves Postpartum Pelvic Floor Function

#### 2.1.1. The Influence of Pregnancy and Childbirth on Female Pelvic Floor Muscles

The female complex pelvic floor support system is composed of pelvic floor muscles and pelvic floor connective tissue. Among them, the pelvic floor muscles mainly include the levator ani muscle and the coccyx muscle; the levator ani muscle is one of the main supporting muscles. The connective tissue of the pelvic floor includes fascia and ligaments, and the muscles of the pelvic floor interact with the connective tissue of the pelvic floor to form a “hanging net,” which together support the pelvic organs in a normal position. The main structure of female pelvic floor muscles is shown in Figure 1.

A series of changes occur in the body of pregnant women: the enlargement of the uterus and the secretion of relaxin will affect the pelvic floor muscles. As the fetus in the womb grows up, the weight of the uterus gradually increases. The resulting waist and abdomen protrude forward and the neutral axis moves forward, which will put pressure on the pelvic floor. Due to the long duration of pregnancy and the continuous and concentrated pressure on the pelvic floor, although the pelvic floor muscle has a certain degree of elasticity, long-term pressure and load will weaken the elasticity of the pelvic floor muscle and impair its toughness. This leads to the deformation of pelvic floor muscle fibers and weakened muscle strength. The pelvic floor muscles cannot support the pelvic organs well, which causes the pelvic organs to leave their normal positions, resulting in a series of pelvic floor dysfunction [10].

RETRACTED

Myogenic injury can induce not only pelvic floor dysfunction but also neurogenic changes. Both acute and chronic changes may cause damage to the pelvic floor muscles. With age and multiple childbirth factors, irreversible changes brought about by pelvic floor injury will gradually aggravate, eventually causing pelvic floor dysfunction [1].

#### 2.1.2. Pelvic Floor Dysfunction Diseases

Pelvic floor dysfunction disease refers to the pathological changes of the pelvic floor tissue structure caused by damage, aging, and other causes of the pelvic floor tissue, which ultimately leads to a series of corresponding organ dysfunction diseases. Its clinical manifestations include lower urinary tract symptoms such as urinary incontinence, lower gastrointestinal symptoms such as pelvic organ prolapse, fecal incontinence, and sexual dysfunction, and a series of symptoms such as pelvic pain. Female pelvic floor dysfunction disease (FPFD) is an important public health problem that affects women's physical and mental health and quality of life. It is very common and is one of the important reasons affecting women's physical and mental health. It is even called “embarrassing social cancer” [11]. Although ABEPS's research and theoretical aspect is correct, this theory needs more practical data to prove it.

#### 2.1.3. Pelvic Floor Rehabilitation Methods

At present, pelvic floor rehabilitation methods include manual massage, pelvic floor muscle exercise (Kegel training method), vaginal dumbbell-assisted pelvic floor muscle training, electrical stimulation therapy, and electrical stimulation combined with biofeedback therapy [12].

Pelvic floor muscle training is widely used due to its convenience in operation, autonomy in choosing time and place, and good intervention effects. The American College of Obstetricians and Gynecologists published in 2009 the clinical practice guidelines for pelvic organ prolapse pointed out that pelvic floor muscle rehabilitation exercise can improve pelvic floor function. For POP with existing symptoms, pelvic floor muscle exercise is recommended as an auxiliary treatment method. The guidelines for diagnosis and treatment of urinary incontinence released by the American Urological Association in 2012 pointed out that women with SUI and mixed urinary incontinence are recommended to exercise pelvic floor muscles as first-line therapy and continue to exercise for more than three months. In 2014, the European Urological Association launched a guideline for urinary incontinence and chronic pelvic pain. The guide pointed out that pelvic floor muscle exercise is better than the nonintervention group in improving female stress urinary incontinence and mixed urinary incontinence. Pelvic floor muscle exercises are used as the first-line treatment for chronic pelvic pain.

RETRACTED

#### 2.1.4. The Physiological Effects of Yoga

During pregnancy and childbirth, the pelvic floor muscles and fascia are excessively stretched, the use of fetal suction, forceps, and other devices in the process of vaginal delivery, and the changes in hormone levels in postpartum women will cause varying degrees of damage to the pelvic floor muscle fibers, resulting in impaired pelvic floor function. A number of studies have shown that adherence to postpartum rehabilitation exercises can effectively restore pelvic floor muscle strength and pelvic floor function [13].

Postpartum yoga exercises are based on the specific conditions of the postpartum women; choosing suitable yoga asanas and loads, with different methods of breathing exercises, meditation, and rest, lets the postpartum women's body and mind be exercised and relaxed so as to achieve the effect of exercising the muscles of the whole body and at the same time promote the recovery of the pelvic floor muscles. Several common yoga exercises to recover pelvic floor muscles are shown in Figure 2.

The 120 postpartum women were divided into a postpartum yoga group and a puerperal exercise group, and they received a 12-week rehabilitation training. The results showed that postpartum yoga was more effective in increasing pelvic floor muscle strength than puerperal exercises; a study on the effect of postpartum yoga exercises on the quality of sexual life of postpartum women showed that postpartum yoga exercises can strengthen the elasticity of the perineum muscles of postpartum women, strengthen the contraction function of the uterus, and prevent a series of symptoms of lower urinary tract prolapse, such as bladder prolapse and vaginal prolapse; moreover, postpartum yoga exercises also have a certain effect on postpartum women's body rehabilitation. In a study on the preventive effect of postpartum yoga on postpartum female urinary incontinence, 360 postpartum women participated in the practice of postpartum yoga. The results show that postpartum yoga combined with pelvic floor muscle training can effectively improve pelvic floor muscle strength, thereby effectively preventing the occurrence of postpartum urinary incontinence, and has a good effect on postpartum women's postpartum body shape and body shaping. Yoga is a form of exercise that requires the participation of body and mind. In the study by Wu Liyan and others, 76 postpartum women were divided into a yoga combined electrical stimulation group and a Kegel exercise group. The results show that yoga combined with electrical stimulation treatment can improve pelvic floor muscle strength more effectively than Kegel exercise alone and has better results in SUI, lumbosacral pain, and sexual arousal disorders [14].

RETRACTED

With the changes in modern people's lifestyles, women's food intake during pregnancy has become more diverse and nutrition is more comprehensive, but the corresponding physical activity has not been kept up. Studies have shown that the incidence of gestational diabetes and hypertension in pregnant women is getting higher and higher. Therefore, women during pregnancy and childbirth should increase their physical activity to maintain the health of themselves and their fetus [15].

#### 2.1.5. The Psychological Effects of Yoga

The mental health of postpartum women has also been the focus of research at home and abroad in recent years. In a study on Hungarians, it was shown that the proportion of pregnant women who are at risk of postpartum depression is about 12% to 16%. Depression during pregnancy is related to the serum hydrocortisone content of pregnant women. If the serum hydrocortisone content is maintained at a high level for a long time, the risk of low birth weight will increase. The American Academy of Obstetrics and Gynecology advocates paying attention to the mental health of postnatal women throughout pregnancy. If you have bad psychological problems, you should take nondrug means to intervene in time.

As one of the oldest traditional methods of health preservation in the world, yoga has its unique charm and characteristics. Compared with other fitness methods that focus on the characteristics of physical exercises, yoga pays more attention to the harmony and unity of the body and mind. Yoga can give full play to its own initiative, mainly through the combination of asanas, consciousness, and breathing; the physical and psychological aspects of the practitioner can be exercised and relaxed, and the movements and asanas of yoga practice are soft and slow; the load and intensity suitable for one's own practice according to one's own situation are chosen; the requirements of different physical conditions of postpartum women are met. Meditation in yoga runs through the entire practice process. Meditation can guide people to focus their attention on beautiful things, eliminate redundant inner thoughts, release stress, relieve fatigue, and relieve depressive emotions [16].

RETRACTED

The physiological mechanism of yoga to relieve depression in postpartum women may include the following aspects: first of all, patients with depression have hypothalamic-pituitary-adrenal (HPA) axis disorders and are accompanied by hypercortisolemia. The results of a randomized controlled experiment showed that yoga can reduce the stress response of the HPA axis and reduce the plasma cortisol level in the blood, so it is believed that yoga may be able to reduce the stress response, thereby reducing the level of depression and treating depression. Secondly, although the regulation mechanism is not clear, studies have confirmed that yoga can regulate neurotransmitters. The influence of norepinephrine, serotonin, dopamine, and other neurotransmitters in the pathogenesis of depression has been widely confirmed. Yoga can increase the level of GABA and dopamine activity in the brain, so it is believed that yoga has a good intervention effect on depression. Finally, patients with depression often show abnormal sleep structures such as increased REM sleep intensity and shallower sleep depth. Yoga can effectively improve the sleep quality of chronic insomnia patients and the elderly. Therefore, it is believed that yoga is helpful in treating the symptoms patients with depression [17].

### 2.2. Asana Recognition Algorithm

In order to better obtain pregnant women's postpartum yoga movements to help improve the rehabilitation of pelvic floor muscle clusters, this article combines asana recognition algorithms to perceive, identify, collect, and help improve yoga asanas. Due to the different sensor types and measurement methods used when recognizing asanas, the magnitude of the detected data may vary greatly. The result will directly cause a certain kind of noise data to dominate because of the large order of magnitude when the algorithm is implemented or to be ignored because the order of magnitude of useful feature data is too small. If these measured data are not preprocessed, it will directly lead to an increase in the error rate of asana recognition. Therefore, before using the original data to identify body poses, the collected pose data must be preprocessed. Commonly used data preprocessing methods are as follows: data normalization; standardization.

#### 2.2.1. Data Normalization

The normalization of data is to uniformly linearly transform the collected data to a new scale. The maximum value on this scale is 1, and the minimum value is 0. The purpose is to eliminate the order of magnitude difference between the data [18]. There are three commonly used data normalization formulas. The first formula is as follows:

(1) $$\begin{array}{c} X_{i}=\frac{X_{i}}{X_{\max}},i\\ =1,2,3\ldots n. \end{array}$$

The second commonly used data is normalized to the maximum and minimum method as follows:

(2) $$\begin{array}{c} X_{i}=\frac{\left(X_{i}-X_{\min}\right)}{\left(X_{i}-X_{\min}\right)},i\\ =1,2,3\ldots n. \end{array}$$

The third method is the mean variance method:

(3) $$\begin{array}{c} X_{i}=\frac{\left(X_{i}-m\right)}{\sqrt{v_{f}}},i\\ =1,2,3\ldots n. \end{array}$$

RETRACTED

#### 2.2.2. Data Standardization

Another preprocessing method in pattern recognition is data standardization; the main purpose is to remove the gap between different units of data. The main method is to calculate the original data according to the original ratio, put them in a relatively small range, and remove the unit of the data to become a dimensionless pure value. There are mainly four methods to achieve linear changes to the original data. The disadvantage is that if new data increase, the maximum and minimum values in the original data will change, and the data standardization process needs to be updated [19]. This method is also called dispersion standardization, and the specific calculation formula is as follows:

(4) $$\begin{array}{c} X_{i}=\frac{\left(X_{i}-X_{\text{min}}\right)}{\left(\text{max}-\text{min}\right)},i\\ =1,2,3\ldots n. \end{array}$$

(5) $$\begin{array}{c} X_{i}=\frac{{\text{log}}_{10}^{X_{i}}}{{\text{log}}_{10}^{\text{max}}},i\\ =1,2,3\ldots n.\\ =1,2,3\ldots n.\\ =1,2,3\ldots n. \end{array}$$

(6) $$\begin{array}{c} X_{i}=\frac{a\text{tan}\left(X_{i}\right)\times 2}{\pi },i\\ =1,2,3\ldots n.\\ =1,2,3\ldots n. \end{array}$$

(7) $$\begin{array}{c} X_{i}=\frac{X_{i}-\mu }{\sigma },i\\ =1,2,3\ldots n. \end{array}$$

In the formula, *μ* is the mean value of the original data and *σ* is the variance.

#### 2.2.3. Asana Feature Extraction

In the field of body recognition, after the sensor collects the signal, it needs to perform feature extraction on the preprocessed raw data. Its purpose is to improve the accuracy and reliability of asana recognition. According to the original acceleration signal collected by the sensor, there are usually three methods to extract asana features: time domain features, frequency domain features, and time-frequency domain features [20].

(1) Time domain characteristics: the time domain feature refers to the extraction of signal characteristics in the time domain, and the main calculation method is the process of statistical analysis of the signal. The main statistical characteristics are mean, variance, maximum, minimum, root mean square, standard deviation, and absolute mean deviation. The maximum value, minimum value, root mean square value, and mean value are used to describe the overall level; variance, standard deviation, and absolute average are used to describe the dispersion of data and differences between data; correlation coefficient is used to describe the association between different variables degree [21].
Average calculation formula is as follows:
  (8) $$\begin{array}{c} \mu =\frac{1}{T}\overset{T}{\underset{i=1}{\sum }}x_{i},i\\ =1,2,3\ldots n, \end{array}$$
where *T* is the length of time to record the original data.
Root mean square value is as follows:
  (9) $$\begin{array}{c} RMS\left(X\right)=\sqrt{\frac{1}{T}\sum_{i=1}^{T}X_{t}^{2}},i\\ =1,2,3\ldots n. \end{array}$$
Variance is as follows:
  (10) $$\begin{array}{c} \sigma =\overset{T}{\underset{i=1}{\sum }}{\left(x_{i}-\mu \right)}^{2},i\\ =1,2,3\ldots n. \end{array}$$
Standard deviation is as follows:
  (11) $$\begin{array}{c} \delta_{X_{i}}=\sqrt{\sum_{i=1}^{T}{\left(x_{i}-\mu \right)}^{2}},i\\ =1,2,3\ldots n. \end{array}$$
Absolute average is as follows:
  (12) $$\begin{array}{c} \text{MAD}\left(X\right)=\frac{1}{T}\overset{T}{\underset{i=1}{\sum }}\left|x_{i}-\bar{X}\right|,i\\ =1,2,3\ldots n. \end{array}$$
Correlation coefficient is as follows:
  (13) $$\begin{array}{c} \text{correlation}\left(X,Y\right)=\frac{\text{cov}\left(X,Y\right)}{\delta_{X}\delta_{Y}}. \end{array}$$
  (14) $$\begin{array}{c} \text{COV}\left(X,Y\right)=E\left[\left(X-\bar{X}\right)\left(Y-\bar{Y}\right)\right]. \end{array}$$
In the formula, cov is the covariance of *X* and *Y* and *δ*_*X*_ and *δ*_*Y*_ are the standard deviations of *X* and *Y*. The calculation of covariance is shown in formula (14).
(2) Frequency domain characteristics: the frequency domain feature is the conversion of the signal, and the feature is extracted from the signal frequency in the frequency domain. It mainly includes fast Fourier transform. The main features extracted include FFT coefficients, signal energy, and entropy in a period of time [22].
Fast Fourier transformation is a fast algorithm of discrete Fourier transform. It uses virtual and real characteristics, symmetry characteristics, and parity characteristics to improve the discrete Fourier transform algorithm to speed up the calculation and introduce butterfly diagrams to assist calculations. Among them, the calculation method of DFT is as follows:
  (15) $$\begin{array}{c} X\left(k\right)=\overset{N-1}{\underset{i=0}{\sum }}x\left(i\right)W_{N}^{ik},k\\ =0,1,2,\ldots N-1, \end{array}$$
  (16) $$\begin{array}{c} x\left(i\right)=\frac{1}{N}\overset{N-1}{\underset{k=0}{\sum }}X\left(k\right)W_{N}^{-ik},i\\ =0,1,2,\ldots N-1, \end{array}$$
  (17) $$\begin{array}{c} W_{N}=e^{-j\frac{2\pi }{N}}. \end{array}$$
Energy mainly describes the energy of the signal in a period of time. The energy of different asanas in the same period of time will vary greatly. The calculation method is mainly that after the signal is transformed by FFT, the amplitude value of each component is squared and then added. According to Paswar's theorem, the signal energy can also be solved in the time domain, and the value of the solution in the time domain is the same as that in the frequency domain [23]. The solution in the frequency domain is as formula (18), and Paswar's theorem is as formula (19).
  (18) $$\begin{array}{c} \text{Energy}\left(X\right)=\frac{\sum_{k=1}^{N}{\left|X\left(k\right)\right|}^{2}}{N}, \end{array}$$
  (19) $$\begin{array}{c} \text{Energy}\left(X\right)=\overset{N}{\underset{i=0}{\sum }}{\left|x\left(i\right)\right|}^{2}=\frac{\sum_{k=1}^{N}{\left|X\left(k\right)\right|}^{2}}{N}. \end{array}$$
(3) Time-frequency domain characteristics: the time-frequency domain feature is mainly to perform wavelet multiscale transformation on the collected signal. Because the wavelet transform can extract the features of the time domain and the frequency domain at the same time and can separately extract the high-frequency and low-frequency characteristics of the signal, it is suitable for the analysis of sports styles. The characteristic of the movement style is that the main feature of the movement is the low-frequency component, so the use of wavelet transform to analyze the low-frequency component can obtain important movement style information [24]. The calculation method of discrete wavelet transform is as follows:
  (20) $$\begin{array}{c} W_{x}\left(j,k\right)=\int_{R}x\left(t\right)\bar{\Psi_{j,k}\left(t\right)}, \end{array}$$
  (21) $$\begin{array}{c} \Psi_{j,k}\left(t\right)=\frac{1}{\sqrt{2^{j}}}\Psi \left(\frac{t}{2^{j}}-k\right). \end{array}$$

RETRACTED

### 2.3. Imaging Examination of the Pelvic Floor

Before imaging examinations are used to diagnose pelvic floor diseases, only clinical assessments are used to determine whether there are structural or functional abnormalities in the pelvic floor organs. More and more clinical studies have shown that clinical evaluation describes superficial anatomy rather than real structural abnormalities, so clinical evaluation alone is not enough to fully evaluate pelvic floor function and anatomy. For example, gynecologists call prolapse of the posterior vaginal wall as “rectocele,” but this clinical manifestation may be caused by at least five different anatomical reasons. Clinical evaluation is usually affected by some unrecognized confounding factors, such as the degree of bladder and rectal filling, the coactivation of the levator ani muscle, and the duration of Valsalva maneuvers [25]. Real-time ultrasound imaging can avoid the expansion of the bladder and rectum through recognition and avoid the coactivation of the levator ani muscle through visual biofeedback so that the examiner can better avoid these situations during the operation. The process of pelvic floor imaging examination is shown in Figure 3:

Before ultrasonography was applied to pelvic floor examination, X-ray examination, as a traditional imaging technique, played an important role in diagnosing pelvic floor lesions. It mainly includes X-ray cystourethrography, cystourethrography, defecography, and other inspection methods under different conditions. The contrast agent is filled in the cavity of the pelvic floor organs for imaging to observe the changes in excretion function and then diagnose the abnormalities of the morphology, movement, and function of various organs.

Ultrasound has been widely used in clinical practice for hundreds of years. Most gynecologists, urologists, and more and more colorectal surgeons have been exposed to the application of ultrasound in clinical work, although most surgeons use transrectal ultrasound rather than transperineal ultrasound. The emergence of B-mode real-time ultrasound makes ultrasound a better choice for examining the pelvic floor organs and functions, whether through the perineum or the vagina. The basic structure and principle block diagram of ultrasound imaging is shown in Figure 4:

A recent study found that the connection between pelvic floor muscle trauma and female POP caused by childbirth is a good example of how imaging can help this article understand the pathophysiology of pelvic floor dysfunction. This allows doctors to do a good job of primary prevention and secondary prevention and allows doctors to carry out effective treatment methods based on imaging studies.

## 3. The Combined Method of Yoga Myoelectrical Stimulation and Traditional Myoelectrical Stimulation Method Control Experiment

### 3.1. Subjects

In this article, 40 parturients who need postpartum pelvic floor rehabilitation were divided into an experimental group and a control group, each with 20 women. The age, parity, and corresponding fetal weight of the experimental group and control group are shown in Tables 1 and 2.

### 3.2. Experimental Method

The experiment divided 40 parturients into two groups, 20 parturients in the experimental group and 20 parturients in the control group. The experimental group performed postpartum pelvic floor rehabilitation experiments using a combination of yoga and myoelectric stimulation for parturients, while the control group only used myoelectric stimulation for postpartum pelvic floor rehabilitation and collected experimental data through pelvic ultrasound examination to analyze the results. In the experiment, data were collected 42 days postpartum and 3 months postpartum. The collected data were resting state, contraction state, and Valsalva state. The results of the two groups of experiments were analyzed by the position of the bladder meridian, the position of the uterus, the position of the rectal ampulla, and the area of the hiatus in the three states.

RETRACTED

### 3.3. Experimental Results

#### 3.3.1. Contracted State

The contraction state is the performance of the muscle in the contraction state. The experiment collected the area of the tears in the contraction state of the parturient 42 days postpartum and 3 months postpartum. The detailed data are shown in Tables 3 and 4.

The experimental result is *P* < 0.05; the experimental data are reasonable. It can be seen from the table that the average area of ruptures in the pelvic floor ultrasound examination in the control group 42 days postpartum was 12.2605 cm^2^, while the average area of ruptures in the pelvic floor ultrasound examination in the experimental group 42 days postpartum was 10.788 cm^2^; in addition, the average area of hiatus in the pelvic floor ultrasound examination in the control group at 3 months postpartum was 11.4805 cm^2^, and the average area of hiatus in the pelvic floor ultrasound examination in the experimental group at 3 months postpartum was 8.9475 cm^2^. This shows that the combination of yoga and myoelectric stimulation has obviously helped postpartum pelvic floor rehabilitation.

#### 3.3.2. Resting State

In order to explore the changes in the position of the bladder meridian, the position of the uterus, the position of the ampulla of the rectum, and the area of the hiatus in the pelvic floor rehabilitation experiment of the parturient by the combination of yoga and myoelectric stimulation in the resting state, the data obtained through pelvic floor ultrasound examination are shown in Figure 5.

It can be seen from the figure that the bladder meridian position in the resting state of the control group women reached an average of 28.3985 mm at 42 days postpartum and an average of 28.015 mm after 3 months; the uterine position reached 37.035 mm on average 42 days postpartum and 35.93 mm after 3 months; the rectal ampulla position reached 17.835 mm on average 42 days postpartum and 19.1605 mm after 3 months; the area of hiatus reached an average of 15.4985 cm^2^ at 42 days postpartum and 15.867 cm^2^ after 3 months. In the experimental group, the position of the bladder meridian in the resting state of the puerpera reached an average of 28.725 mm at 42 days postpartum and an average of 29.74 mm after 3 months; the position of the uterus reached an average of 34.995 mm at 42 days postpartum and an average of 39.54 mm after 3 months; the rectal ampulla position reached an average of 21.15 mm on 42 days postpartum and an average of 22.82 mm after 3 months; the hole area reached an average of 14.4 cm^2^ at 42 days postpartum and an average of 13.5355 cm^2^ after 3 months. Comprehensive data analysis can be obtained through the method of yoga combined with myoelectric stimulation, the rehabilitation of the bladder meridian and rectal ampulla is significantly better than the method of only using myoelectric stimulation. Moreover, only using the myoelectric stimulation method may lead to failure of the uterine position reset, and the combination of yoga and myoelectric stimulation can very effectively recover the uterine position. Furthermore, only using myoelectric stimulation has little effect on the slit area, but the combination of yoga and myoelectric stimulation can quickly recover the slit area.

RETRACTED

#### 3.3.3. State of Valsalva

Valsalva is simple, practical, and noninvasive and has been used clinically for a long time. In the Valsalva test, the patient is forced to shut down and perform an exhalation maneuver. In other words, close the glottis after taking a deep breath, enforce the exhalation action, fight with the closed laryngeal lid during exhalation, and affect blood circulation and autonomic nerve function. By increasing the state of intrathoracic pressure, clinical physiology examination for the purpose of diagnosis and treatment is achieved.

By increasing the pressure in the chest cavity, the amount of blood returning from the veins is greatly reduced; the vagus nerve is gradually excited. (1) In the case of the paroxysmal upper ventricular artery, use Valsalva to excite the labyrinth nerve and end the upper ventricular artery; (2) hypertrophic cardiomyopathy obliterans, at the same time, due to the effect of Valsalva, reduces the amount of blood returned to enhance dullness, used to judge dullness; (3) mitral valve prolapse causes mitral valve regurgitation, and the dullness is enhanced by Valsalva action; (4) due to the effect of Valsalva, the murmur of the left and right heart will generally be weakened, and the narrow murmur under the idiopathic hypertrophy will increase. Clinicians often use this action to determine the nature and source of noise. Valsalva cannot be used for too long. If it is too long, cerebral blood flow and coronary blood flow will decrease. Therefore, this article collected the ultrasound examination data of the position of the bladder meridian, the position of the uterus, the position of the ampulla of the rectum, and the area of the hiatus and the pelvic floor in the Valsalva state, as shown in Figure 6.

RETRACTED

It can be seen from the figure that the position of the bladder meridian in the Valsalva state of the control group of women reached −3.26 mm on average at 42 days postpartum and −3.225 mm after 3 months; the uterine position reached an average of 12.7515 mm at 42 days postpartum and 14.195 mm after 3 months; the rectal ampulla position reached an average of −6.585 mm on 42 days postpartum and an average of −8.435 mm after 3 months; the hole area reached an average of 24.4415 cm^2^ at 42 days postpartum and an average of 23.203 cm^2^ after 3 months. In the experimental group, the position of the bladder meridian in the Valsalva state of the experimental group reached an average of 6.465 mm at 42 days postpartum and an average of 11.805 mm after 3 months; the position of the uterus reached an average of 22.485 mm at 42 days postpartum and an average of 28.565 mm after 3 months; the rectal ampulla position reached 3.81 mm on average 42 days after delivery and 10.535 mm on average after 3 months; the hole area reached an average of 20.908 cm^2^ at 42 days postpartum and 17.5035 cm^2^ after 3 months. Comprehensive data analysis can be obtained, only using electromyographic stimulation method in the Valsalva state bladder meridian position and rectal ampulla position will reach a negative number, the combined method of yoga and myoelectric stimulation reached 6.465 mm at 42 days postpartum at the bladder meridian position in Valsalva state and recovered to 11.805 mm after 3 months; the rectal ampulla position reached 3.81 mm 42 days postpartum and recovered to 10.535 mm after 3 months. The rehabilitation degree of the parturient area of the parturient who was trained by the combination of yoga and myoelectric stimulation was much better than that of only using the myoelectric stimulation method.

## 4. Yoga's Analysis of Maternal Physical and Mental Health

After ten weeks of yoga practice, the independent sample *t*-test was performed on the physical fitness indicators of the experimental group and the control group. The statistical results are shown in Table 5.

It can be seen from Table 5 that the effect of yoga on postpartum women's physical function recovery is still very obvious, and the difference between the experimental group and the control group is obvious. As shown in Table 5, the difference in chest circumference, vital capacity difference, and *P* value of sitting body forward bending between the experimental group and the control group are all less than 0.01, and there is a significant difference; the *P* values of vital capacity, seated forward flexion difference, grip strength, and closed-eye single foot difference were all less than 0.05, and there were differences. Although the difference in grip strength and the *P* value of closed eyes and single foot stand did not show any difference, it is reflected in the numerical value that the data of the experimental group is significantly higher than that of the control group. Therefore, yoga exercise has a promoting effect on improving the body function and state of the parturient.

RETRACTED

The SCL-90 psychological scale survey was conducted on the experimental subjects before and after the experiment, and the experimental data results are shown in Figure 7.

It can be seen from the figure that the ratio of the normal value after the experiment is higher than the ratio of the value before the experiment. In particular, psychological indicators such as anxiety and paranoia were higher than normal before the experiment, but they all returned to the normal range under the intervention of yoga. The psychological test indicators such as depression and hostility decreased compared with those with higher scores before the experiment. These results show that under the intervention of yoga practice, the mental health of the parturient is improved. In order to make the experiment more scientific, this article also compares and analyzes the mental health indicators of normal people across the country. The results of the experiment are shown in Figure 8.

It can be seen from the figure that although there is no significant difference in the values of the mental health indicators of the pregnant women before and after the experiment, they have all declined. Moreover, compared with the data before the experiment, the values of various factors after the experiment are closer to the normal adult data of the whole country. This also illustrates the curative effect of yoga intervention on the mental health rehabilitation of parturients.

## 5. Conclusions

This article mainly studies the influence of yoga on postpartum pelvic floor rehabilitation. This article understands the methods of postpartum pelvic floor rehabilitation for parturients and combines yoga to improve the methods of pelvic floor rehabilitation for parturients. Postpartum yoga is identified and improved by the body position recognition algorithm, aiming to explore which yoga posture can best improve the speed of maternal pelvic floor recovery. Therefore, this article designed a set of controlled experiments to perform pelvic ultrasound examinations on the 42 days and 3 months postpartum of parturients. Through experimental comparison, it is concluded that in the resting state, contracted state, and Valsalva state, the position of the bladder meridian, the position of the uterus, and the position of the rectal ampulla of the parturient women have significantly recovered compared with the traditional electromyography treatment. In addition, the average area of hiatus in the pelvic floor ultrasound examination in the control group 42 days postpartum was 12.2605 cm^2^, while the average area of the hiatus in the pelvic floor ultrasound examination in the experimental group 42 days postpartum was 10.788 cm^2^. In the control group, the average area of hiatus in pelvic floor ultrasound examination at 3 months postpartum was 11.4805 cm^2^. In the experimental group, the average area of the hiatus in the pelvic floor ultrasound examination at 3 months postpartum was 8.9475 cm^2^, and yoga had a very significant improvement on the physical indicators and mental health of the postpartum women.

RETRACTED

## Figures and Tables

**Figure 1:** Female pelvic floor muscle structure.

**Figure 2:** Several common yoga exercises to rehabilitate the pelvic floor muscles.

**Figure 3:** The process of pelvic floor imaging examination.

**Figure 4:** Basic structure principle of ultrasound imaging.

**Figure 5:** Comparison of experimental results at rest. (a) Results of pelvic floor ultrasound examination in the control group. (b) Bottom ultrasound examination results of the experimental group.

**Figure 6:** Comparative experimental results in Valsalva state. (a) Results of pelvic floor ultrasound examination in the control group. (b) Results of pelvic floor ultrasound examination in the experimental group.

**Figure 7:** Numerical ratio of mental health indicators of parturients before and after the experiment. (a) Before the experiment. (b) After the experiment.

**Figure 8:** Comparison of mental health indicators of parturients before and after the experiment and the national norm. (a) Before the experiment. (b) After the experiment.

**Table 1:** Details of maternal data in the control group.

Serial number	Age	Parity	*P*
1	37	2	0.0014
2	29	1	0.0023
3	31	2	0.0011
4	31	2	0.0015
5	29	1	0.001
6	32	1	0.0023
7	30	1	0.0016
8	33	1	0.0025
9	28	1	0.0026
10	33	1	0.0014
11	37	1	0.001
12	36	2	0.0024
13	23	1	0.0016
14	32	2	0.002
15	31	2	0.0014
16	37	1	0.0021
17	29	1	0.0017
18	29	2	0.0016
19	37	2	0.0018
20	29	1	0.001

**Table 2:** Details of maternal data in the experimental group.

Serial number	Age	Parity	*P*
1	28	1	0.0012
2	32	1	0.001
3	38	1	0.0028
4	36	2	0.003
5	32	1	0.0024
6	22	1	0.0018
7	35	2	0.0014
8	29	1	0.002
9	36	2	0.0012
10	32	2	0.0025
11	30	1	0.0011
12	30	1	0.0024
13	29	1	0.0018
14	28	1	0.0014
15	28	1	0.0011
16	25	1	0.0029
17	31	1	0.0024
18	28	2	0.0018
19	28	1	0.0026
20	28	1	0.0027

It can be seen from the table that the average age distribution of parturients (*P* < 0.05) can be used as experimental objects.

RETRACTED

**Table 3:** Results of ultrasound examination of the pelvic floor under contraction in the control group.

Serial number	Hole area (cm^2^)		*P*
	42 days postpartum	3 months postpartum	
1	13.59	14.7	0.0026
2	11	9	0.0026
3	14.82	11.5	0.0027
4	8.59	8.09	0.0016
5	10.86	10.73	0.0019
6	10.92	9.6	0.0013
7	14.75	13.71	0.0022
8	12.52	14.28	0.0016
9	9.04	9.03	0.0026
10	16	13	0.002
11	9.92	11	0.0024
12	17	17	0.0021
13	14	9	0.0026
14	10	8.6	0.0023
15	16	12.4	0.0024
16	15.8	14.4	0.0012
17	10	13	0.0025
18	10.76	11.17	0.003
19	16.01	11.26	0.0011
20	10	11.96	0.0014

**Table 4:** Results of ultrasound examination of the pelvic floor under contraction in the experimental group.

Serial number	Hole area (cm^2^)		*P*
	42 days postpartum	3 months postpartum	
1	10.48	9.49	0.0029
2	14.12	9.35	0.0029
3	13.17	12.55	0.0023
4	12.69	8.25	0.002
5	10.44	8.17	0.002
6	12.46	9.87	0.0013
7	9.57	8.45	0.002
8	15.5	9.96	0.0022
9	9.31	7.81	0.003
10	10.18	6.7	0.002
11	10.96	8.85	0.0014
12	9.33	7.82	0.0016
13	6.66	8.18	0.001
14	9.09	9.75	0.0024
15	9.21	9.23	0.0011
16	8.44	8.73	0.0015
17	7.72	7.53	0.0016
18	12.69	11.9	0.0011
19	10.1	9.8	0.0011
20	13.64	10.06	0.0024

**Table 5:** Comparison of physical fitness indexes between the experimental group and the control group after the experiment.

Index	Control group	Test group	*P*
Poor bust	3.38 ± 0.62	4.40 ± 1.03	0.003 ^*∗∗*^
Vital capacity	744 ± 274	2853 ± 461	0.02 ^*∗*^
Sitting forward bending	13.91 ± 8.22	17.93 ± 4.35	0.01 ^*∗∗*^
Grip	23.99 ± 2.69	26.63 ± 3.82	0.04 ^*∗*^
Close eyes and single foothold	29.60 ± 21.89	6.01 ± 3.97	0.03 ^*∗*^

## Data Availability

No data were used to support this study.

## References

[1] Meng X., Feng L., Chen H. (2021). Just-in-Time human gesture recognition using WiFi signals. *Chinese Journal of Electronics*.

[2] Zhou F., Li X., Wang Z. (2020). Efficient high cross-user recognition rate ultrasonic hand gesture recognition system. *IEEE Sensors Journal*.

[3] Modanwal G., Sarawadekar K. (2018). A robust wrist point detection algorithm using geometric features. *Pattern Recognition Letters*.

[4] Zadghorban M., Nahvi M. (2018). An algorithm on sign words extraction and recognition of continuous Persian sign language based on motion and shape features of hands. *Pattern Analysis & Applications*.

RETRACTED

[5] Bhattacharyya S. . (2018). Optimization of a HMM-Based Hand Gesture Recognition System Using a Hybrid Cuckoo Search Algorithm. *Hybrid metaheuristics for image analysis*.

[6] Dunleavy K., Kava K., Goldberg A. (2016). Comparative effectiveness of Pilates and yoga group exercise interventions for chronic mechanical neck pain: quasi-randomised parallel controlled study. *Physiotherapy*.

[7] Cheung C., Wyman J. F., Bronas U., McCarthy T., Rudser K., Mathiason M. A. (2017). Managing knee osteoarthritis with yoga or aerobic/strengthening exercise programs in older adults: a pilot randomized controlled trial. *Rheumatology International*.

[8] Park Y.-H., Kim J. (2018). The influence of yoga Instructor’s image and non-verbal communication on instructors trust and intimacy of yoga exercise participants. *Korean Journal of Sports Science*.

[9] Bhatia T., Mazumdar S., Wood J. (2016). A randomised controlled trial of adjunctive yoga and adjunctive physical exercise training for cognitive dysfunction in schizophrenia. *Acta Neuropsychiatrica*.

[10] Mathersul D. C., Rosenbaum S. (2016). The roles of exercise and yoga in ameliorating depression as a risk factor for cognitive decline. *Evidence-based Complementary and Alternative Medicine*.

[11] Saudia B. E. P., Kisid K. M., Andarini M., Mustofa E. (2018). The effects of yoga exercise on lipid peroxidation and antioxidant status in pregnant women. *Indian Journal of Medical Specialities*.

[12] Kim H.-K., Kim S.-H., Kim Y.-P. (2017). The effect of Yoga exercise on daily-living fitness and aging hormone in elderly women. *Korean Journal of Sports Science*.

[13] Li D. J., Li Y. Y., Li J. X., Fu Y. (2018). Gesture recognition based on BP neural network improved by chaotic genetic algorithm. *International Journal of Automation and Computing*.

[14] Wei X., Wang M., Xiao L. (2017). Research of human gesture recognition algorithm based on multi-layer perceptron. *AIP Conference Proceedings*.

[15] Ghosh D. K., Ari S. (2016). On an algorithm for Vision-based hand gesture recognition. *Signal, Image and Video Processing*.

[16] Li F., Fei J. (2019). Gesture recognition algorithm based on image information fusion in virtual reality. *Personal and Ubiquitous Computing*.

[17] Jiang D., Li G., Sun Y., Kong J., Tao B. (2019). Gesture recognition based on skeletonization algorithm and CNN with ASL database. *Multimedia Tools and Applications*.

[18] Hyun J. H., Kang D. S. (2017). A study on hand gesture recognition algorithm for immersive interface implementation based on DTV and HNN. *The Journal of Korean Institute of Information Technology*.

[19] Hwang D. H., Jang K. S. (2017). Hand-Gesture recognition using concentric-circle expanding and tracing algorithm. *Journal of the Korea Institute of Information and Communication Engineering*.

RETRACTED

[20] Zhang W., Smith M. L., Smith L. N., Farooq A. (2016). Gender and gaze gesture recognition for human-computer interaction. *Computer Vision and Image Understanding*.

[21] Xie R., Cao J. (2016). Accelerometer-based hand gesture recognition by neural network and similarity matching. *IEEE Sensors Journal*.

[22] Jiye K., Jong-Il (2017). HOG-HOD algorithm for recognition of multi-cultural hand gestures. *Journal of Korea Multimedia Society*.

[23] Chongshan L., Ting Z., Chengyuan L. (2017). An improved otsu’s thresholding algorithm on gesture segmentation. *Journal of Advanced Computational Intelligence and Intelligent Informatics*.

[24] Mo T., Sun P. (2020). Research on key issues of gesture recognition for artificial intelligence. *Soft Computing*.

[25] Ebrahimi M., Guilan-Nejad T. N., Pordanjani A. F. (2017). Effect of yoga and aerobics exercise on sleep quality in women with Type 2 diabetes: a randomized controlled trial. *Sleep Science*.

